This article has been retracted.

# Research Progress on the Mechanism of Right Heart-Related Pulmonary Edema

**DOI:** 10.1155/2022/8947780

**Published:** 2022-08-03

**Authors:** Yiran Li, Xiaoqiang Wang, Ruiqing Zong, Feixiang Wu, Hai Lin

**Affiliations:** ^1^Department of Intensive Care Medicine, Eastern Hepatobiliary Surgery Hospital, The Third Affiliated Hospital of Naval Medical University, Shanghai 200438, China; ^2^Department of Anesthesiology, Renji Hospital, Shanghai JiaoTong University School of Medicine, Shanghai 200127, China; ^3^Department of Emergency, Maanshan People's Hospital, Maanshan 243000, China

## Abstract

**Objective:**

To investigate the mechanisms underlying the development of right heart-associated PE.

**Background:**

Right heart-related pulmonary edema (PE) refers to PE resulting from impaired right heart function caused by primary or secondary factors, which is common in critically ill patients. Although the clinical manifestations of different types of right heart-related PE are similar, the pathophysiological changes and treatment methods are significantly different. According to the hemodynamic mechanism, right heart-related PE is primarily classified into two types. One is the increase of right heart flow, including extravascular compression, intravascular compression, cardiac compression, and cardiac decompression. The other type is the abnormal distribution of pulmonary circulation, including obstruction, resistance, pleural decompression, or negative pressure. With the development of hemodynamic monitoring, hemodynamic data not only help us understand the specific pathogenesis of right heart-related PE but also assist us in determining the direction of therapy and enabling individualized treatment. *Summary.* This article presents a review on right heart-associated PE, with a perspective of hemodynamic analysis, and emphasizes the importance of right heart function in the management of circulation. Understanding the mechanism of right heart-associated PE will not only aid in better monitoring right heart function but also help intensivists make a more accurate identification of various types of PE in the clinic.

## 1. Introduction

Acute pulmonary edema (PE) refers to fluids infiltrating from the pulmonary capillaries into the pulmonary interstitium and alveoli, which affects gas exchange and causes cough, foamy sputum, dyspnea, hypoxemia, and other syndromes [1]. It is one of the common critical illnesses. Based on the mechanism of occurrence, PE is divided into two categories. One is cardiogenic PE (CPE), also known as hydrostatic PE, which is often caused by various reasons for acute decompensated heart disease causes [2]. It is the serious stage of heart exhaustion. The other category is noncardiogenic PE, which is caused by other diseases such as acute lung injury, sepsis, allergies, and high-altitude hypoxia, which increases capillary permeability, resulting in PE [3].

With further understanding of hemodynamics, we have gradually realized that right heart-related PE is as common as PE associated with the left heart [4]. Right heart failure occurs when the right ventricular function is decompensated. With a sharp decrease in stroke volume, pulmonary artery resistance increases, thereby promoting the occurrence of PE. A mismatch between right- and left-sided filling pressures result in hemodynamic abnormalities, and the PE will be further aggravated. Earlier, our understanding of the right heart was derived from the invasive monitoring of the pulmonary artery catheter, and its clinical application was limited [5]. In recent years, noninvasive monitoring of hemodynamics, such as by ultrasound, has been increasingly applied in clinical practice [6, 7]. In December 2017, the collaborative group of severe hemodynamic therapy published an expert consensus on the management of severe right cardiac function [8], which clearly indicated that the right heart is a status of the theory of critical care medicine and critical care hemodynamics and that the understanding of the right heart is a part of the diagnosis and treatment of critical care disease. Hemodynamics is concerned with the movement of blood. The movement of blood is spread throughout the body, linking the body's tissue cells and organs together like a network. The pattern of blood movement in the body is different from the general fluid dynamics, which is influenced by various factors such as physiology and pathology. As our understanding of hemodynamics has improved, our assessment of right heart function has become more refined, and we have gained further insight into the relationship between the right heart and CPE. Hemodynamic parameters such as blood pressure, cardiac output, and arterial oxygen content directly reflect the changes that occur in a specific part of the body and their degree, thereby hinting at the treatment method to be used and allowing optimization of the entire treatment process. In hemodynamic therapy, the direction of the treatment strategy and the quantitative adjustment of the treatment method are integrated throughout the treatment process. This process also facilitates a new understanding of the disease process, which is timelier in detecting the cause of PE and more responsive to the actual needs of the organism.

## 2. Classification and Mechanism of Right Heart-Related Pulmonary Edema

According to the hemodynamic mechanism, PE associated with the right heart is primarily divided into two categories. One is the increase of right heart flow, including extravascular compression, intravascular compression, cardiac compression, and cardiac decompression. The other is the abnormal distribution of pulmonary blood flow, including obstruction, resistance, pleural decompression, or negative pressure. Using such classification, the direction of treatment is determined, and simple symptomatic treatment is avoided. Quantitative adjustments make the implementation of treatment methods more accurate due to the mastery of the intensity of treatment. This review is intended to discuss the pathogenesis of right heart-associated PE in two major categories and summarize the key points (Table 1), with an anticipation of providing new ideas for the treatment of right heart-associated PE.

### 2.1. Increased Right Heart Flow

#### 2.1.1. Extravascular Compression

Peripheral venous contraction is caused by various reasons, and hence, the amount of blood returning to the heart is increased significantly in a short time, which is often accompanied by increased cardiac afterload. Left ventricular dysfunction is more likely to occur. It primarily refers to exercise-induced PE (EIPE), which is closely related to activities such as swimming, marathon, and extreme sports [9–11]. The primary pathophysiology of EIPE is arterial and venous vasoconstriction, which results in the centripetal distribution of blood flow and increased cardiac load before and after. Swimming-induced PE (SIPE), also known as immersion PE, occurs in people that practice water sports such as swimming and snorkeling, and hence, its name was first reported in divers in 1981 [12]. Regarding its pathogenesis, when the body is in the water, the peripheral volume of blood vessel pressure increases, leading to the redistribution of blood in the chest cavity, venous reflux, and increased biventricular preload. Especially for triathletes, the tight neoprene diving suits further aggravate this redistribution, which may cause obvious hemodynamic changes. When people are immersed in motionless water, their central venous pressure increases by 12–18 mmHg and their stroke output becomes>25% [13]. Exercise in cold water can increase the average pulmonary arterial pressure and pulmonary artery wedge pressure, resulting in PE. Some studies have demonstrated that increased hydrostatic pressure can cause microscopic fracture of the blood-gas barrier membrane, which is known as capillary stress failure, and thus patients with SIPE will present hemoptysis [14, 15]. When a patient has SIPE, he/she must get out of the water immediately, remove the tight diving suit or swimsuit, and move into a warm environment. Supportive therapies may be administered on a case-by-case basis, including oxygen, diuretics, and beta-2 receptor agonists. Vasodilators such as sildenafil and dihydropyridine calcium channel blockers can prevent SIPE [16].

In the case of high-altitude PE (HAPE), the person's pulmonary arterial pressure and pulmonary blood volume increase rapidly due to hypoxia when he/she rapidly moves from plains to plateau, and then the liquid in the capillary seeps into the pulmonary interstitium and alveolus, causing PE. Pulmonary hypertension is characterized by a rapid increase after entering the plateau for several hours. The mean pulmonary arterial pressure of patients with HAPE is between 36 and 51 mmHg, whereas the pulmonary capillary pressure is between 20 and 26 mmHg. Endothelin-1 has a powerful function of constricting pulmonary vessels, and high levels of endothelin-1 have been shown in patients susceptible to HAPE. Under the induction of a plateau environment, an elevated plasma endothelin-1level is directly related to pulmonary hypertension [17]. Some studies have also suggested that the increase in oxidative stress-free radicals can reduce the synthesis and release of NO in the lungs in the case of hypoxia, and NO can dilate pulmonary blood vessels and cause hypoxia, thereby strengthening pulmonary vasoconstriction [18, 19]. HAPE is associated with extravascular compression, but not primary.

Extravascular compression is also related to neuroendocrinology, including various sympathetic catecholamine storms, application of various vasopressor drugs, and endocrine tumors [20, 21]. Neurogenic PE (NPE) is a potential complication of diseases of the central nervous system such as cerebral hemorrhage, uncontrolled seizures, coma, brain tumors, and neurosurgery [22]. Its etiology is presumed to be an intense discharge due to a wide range of central nervous system diseases [23]. Pheochromocytoma can cause life-related PE, which can be rapidly fatal but is clinically uncommon. It has been reported that cardiogenic shock and myocardial infarction cannot be ruled out in patients with acute PE. These patients are often treated with high-dose myocardial inotropic drugs and intra-aortic balloon counter pulsation. To exclude abdominal aortic aneurysm, abdominal CT revealed the presence of a 6-cm mass in the right adrenal gland. After reducing the dosage of positive inotropic drugs, the levels of 24 h urine catecholamine and norepinephrine remained elevated, thus confirming pheochromocytoma. After tumor resection and drug control for a week, the cardiac function gradually returned to normal. Therefore, it is necessary to consider the possibility of pheochromocytoma when PE and shock are difficult to explain [24]. The hemodynamic mechanism of NPE is primarily pulmonary circulation overload and pulmonary vasoconstriction. Intracranial pressure increases sharply after central nervous system damage, and then the cerebral blood flow decreases. Simultaneously, due to hypothalamus dysfunction, the inhibitory effect of the nuclear level before the eye and the “edema center” of the hypothalamic tail is decreased, and both can result in sympathetic nervous excitement. Catecholamine levels in the circulating blood increase suddenly, causing vasoconstriction of the systemic circulation and pulmonary circulation. Increased blood pressure in systemic circulation can cause a large amount of blood flow from the systemic circulation to the pulmonary circulation, which causes an increase in pulmonary vascular volume. When a large amount of blood from the pulmonary circulation enters into the low-pressure area, the pulmonary vascular hydrostatic pressure increases and NPE develops [2]. Furthermore, evidence suggests that NPE can be reduced or avoided by the administration of both sympathetic blockers and adrenaline receptor blockers.

#### 2.1.2. Intravascular Compression

Intravascular compression refers to the relative or absolute overload of blood vessel volume. When rapid capacity load occurs, the proximal cardiac artery and vein short-circuit causes a significant increase in the right cardiac load, which occurs more frequently in people with left cardiac dysfunction. Clinically, fluid overload PE could be easily detected in patients with hypoxia, pneumonia, anemia, cardiac or renal insufficiency, anesthesia, cardiac surgery, and low plasma protein. When the infusion is excessive and very rapid, it can easily induce PE. Moreover, when a large amount of fluid input is used to maintain effective blood volume of patients with shock and severe trauma in the ICU, the combination of powerful vasoconstrictor drugs such as norepinephrine can promote more systemic blood into the lower pressure of pulmonary circulation, increasing pulmonary capillary pressure. The fluid leaks out into the alveoli, and PE develops [25]. Studies have found that several cases of CPE also contain water and sodium retention and fluid overload caused by abnormal fluid distribution [26]. Regarding the mechanism of occurrence, pulmonary capillary wedge pressure increases in both CPE and pure liquid overload PE; however, the occurrence of PE is related to the increased rate of pulmonary capillary hydrostatic pressure. Due to the continuous progression of heart failure, CPE occurs, and thus pulmonary capillary hydrostatic pressure in patients with CPE is often higher than that in patients with liquid overload PE.

For evaluating the circulatory function in this type of PE, ultrasound can be used to monitor the diameter of the inferior vena cava, and respiratory variability can be used to assess fluid reactivity and volume load status; however, this indicator is more susceptible to right heart function, pulmonary circulation resistance, and right heart preload. It should be combined with clinical comprehensive judgment [27]. Due to a variety of factors, central venous pressure as an indicator of early cardiac preload assessment is often unable to accurately reflect the cardiac preload. Pulmonary wedge pressure is considered to be the gold standard for the diagnosis of acute PE. When pulmonary wedge pressure is > 18 mmHg, it indicates that PE is caused by excessive volume overload. The pulmonary thermodilution method consists of injecting ice-cold physiological saline into the central vein, detecting it using a thermistor at the end of the aorta (femoral or radial artery) catheter, and plotting a thermodilution curve. When edema is present in the lungs, the arterial thermosensitive probe monitors increased thermal dilution (fluid warming); this indicator loss can be used to quantify extravascular lung water. Ultrasonic cardiac output monitor is a noninvasive cardiac output monitoring technology that can judge the capacity load indirectly. Regarding its principle, when patients passively lift their legs, the return blood volume changes, which cause changes in blood flow velocity in the outflow tract of the left ventricle. If the stroke volume increases at this time, the patient's fluid capacity is insufficient, and vice versa [28].

#### 2.1.3. Cardiac Pressurization

Ventricular interaction is one of the important mechanisms and bases of hemodynamic changes and corresponding adjustments. The management of hemodynamics requires a complete understanding of ventricular interactions. Regardless of the adjustment of volume, cardiac function, or post load, it is important to consider the interaction between the left and right ventricles and the effect of the corresponding treatment on the two ventricles. Both the left and right ventricles are interdependent and interact. Changes in volume and pressure of one side of the ventricle or changes in myocardial hardness and contractile force of one side of the ventricle will affect the other ventricle. The prominent effect of right-sided heart failure on left-sided heart function is that the left heart filling is affected, and the left ventricular diastole is limited. The left ventricular filling pressure is increased, leading to the increase of pulmonary water outside the blood vessels, resulting in PE. The right heart function plays a vital role in the formation mechanism of PE, which can limit the left heart diastole through the interaction between the left and right ventricles. When the change of right heart flow exceeds the matching range of pulmonary circulation and left heart adaptability, PE increases.

Cardiac vasopressor PE can be divided into two conditions. First, the left heart function is weakened by left heart infarction or left heart stress cardiomyopathy, due to which the left and right heart functions do not match. The second condition is the enhancement of right cardiac systolic activity, which often occurs in left cardiac dysfunction, due to which the left and right cardiac functions do not match. Furthermore, close attention should be paid to the shunt between the right and left heart. In addition to congenital heart disease, new left-to-right shunt should be excluded from severe diseases. For instance, if patients with myocardial infarction are complicated with ventricular septal perforation, a new left-to-right shunt will cause a sudden increase in the volume load of the right heart, which causes PE. Through cardiac ultrasound, we can correctly evaluate the functions of the left and right heart, thereby maintaining appropriate preload status, avoiding insufficient capacity, inhibiting the high blood pressure that has satisfied perfusion under the sufficient cardiac output, controlling the ventricular rate in a stable range, and maintaining the circulation of the left and right heart and lungs in a relatively stable state.

#### 2.1.4. Cardiac Decompression

Cardiac decompression refers to the decompression of the pericardium or pleural cavity, resulting in increased pulmonary blood flow, causing PE. PE is more likely to occur in patients with left heart obstruction due to a rapid reduction of pericardial pressure and an increase in short-term cardiac blood volume and right cardiac output [29]. When patients, whose blood flow is blocked have pericardial effusion, pulmonary vein blood flow is also blocked. The volume of blood flowing back to the right heart is also reduced when the fluid is accumulated. The volume of blood, that is, injected into the pulmonary artery by the right heart is also reduced. At this time, although the pulmonary vein hardly returns the blood to the left atrium and the lungs are congested, the volume of blood injected by the right heart into the pulmonary arteries decreases. This does not cause pulmonary congestion and edema. When effusion draws out excessive blood very rapidly, the heart press against pressure removes. Blood is highly circumfluent. The blood that shoots into the pulmonary artery is a short time increase, and pulmonary organization has a lot of blood siltation in a short time, which brings about acute PE. Clinical management principles include sedation, oxygen, reduction of venous reflux, and rapid diuretics at this time. If the duration of the cardiac tamponade is longer, the myocardium has different degrees of injury, i.e., atrophy. Extraction of excessive fluid to remove the cardiac tamponade can result in acute expansion of the heart or a rapid increase in the amount of blood flowing back. Left atrial pressure increases, and pulmonary capillary pressure increases. Plasma penetrates into the tissue gap or alveolus, which causes acute PE.

### 2.2. Abnormal Pulmonary Circulation

#### 2.2.1. Obstructive Factors

Due to a few reports on PE occurring after pulmonary embolism, the clinical understanding is insufficient. The presence of edema may mask the timely diagnosis and management of pulmonary embolism. Pulmonary embolism results in decreased pulmonary circulation area and overperfusion in nonembodied areas, which may be one of the primary factors of PE. In animal experiments, embolization or balloon blockade of pulmonary vessels could induce leakage of nonembodied areas and PE [30]. Similar changes occur in patients with clinical pulmonary embolism [31]. Hultgren proposed the perfusion mechanism, which is used to elucidate the hemodynamics of HAPE, which can also be used to explain the occurrence of pulmonary embolism-associated PE. Yuceoglu, who investigated lung embolism-related PE, found that 51% of patients with pulmonary embolism developed PE [32]. The majority of these patients had a coronary heart disease basis, and those without coronary heart disease had less probability to develop PE. This indicates that this type of perfusional PE is more likely to occur in patients with left ventricular diastolic or systolic dysfunction. However, PE in the normal perfusion area can still occur in some patients with pulmonary embolism, who have no previous history of heart disease and no clinical left heart disorder [33]. These patients can be easily misdiagnosed with PE, ignoring the potential real cause. Cardiopulmonary ultrasound can rapidly identify such patients [34].

#### 2.2.2. Resistance Factors

Several factors under pathophysiological conditions can lead to changes in pulmonary circulatory resistance, resulting in a redistribution of pulmonary blood flow and imbalance of pulmonary circulatory blood flow and pressure distribution, thereby causing regional over perfusion and increased heterogeneity of lung water. Hypoxia-induced HAPE, which is characterized by pulmonary vasoconstriction, is a typical representative of PE associated with acute pulmonary circulation resistance changes. Although most studies suggest that HAPE is associated with damaged endothelium and alveolar epithelium caused by inflammatory responses under hypoxic conditions, which involve several pathways and mediators, including hypoxia-inducible factor, vascular endothelial growth factor, endothelin-1, and inducible nitric oxide synthase, and also involving sodium channels that regulate water transport, Na-K-ATPase, and aquaporin, pulmonary hemodynamic changes and higher hydrostatic pressure play a vital role in the acute and rapid progression of HAPE [35–38]. The initial alveolar protein and red blood cells appear before the inflammatory mediators in the early stage of HAPE, suggesting that the initial movement is the mechanical damage (stress) of the pulmonary capillary bed caused by the change in pulmonary circulation pressure. Visscher proposed that pulmonary vasculature show heterogeneity shrinkage during hypoxia [39]. This change reduces blood flow in the vasoconstriction area, whereas the non-vasoconstriction area is subjected to relatively large blood flow and pressure, which causes damage of mechanical stress and induction of HAPE. Pulmonary artery catheter and isotope-labeled transferrin were used to examine patients with HAPE. Pulmonary arterial pressure, capillary pressure, and transcapillary leakage were significantly increased in the early stage of hypoxic exposure, suggesting that the early increase of lung water and the increase of hydrostatic pressure in such patients are highly closely related [17]. Due to body position and gravity, the pulmonary blood flow of the body exhibits an inhomogeneous distribution, and hypoxia can aggravate the spatial heterogeneity of pulmonary blood flow, which leads to higher pulmonary circulation resistance, higher pulmonary arterial pressure, and higher pulmonary capillary embedding. The occurrence of HAPE is closely related to this change, and the heterogeneity is related to the distribution of vascular smooth muscle, the response of smooth muscle to hypoxia, and the presence of nonmacular arterioles [40, 41].

Monitoring of pulmonary arterial pressure in HAPE-susceptible populations by echocardiography revealed that pulmonary arterial pressure was more vulnerable to escalation in these populations in high-altitude areas than in no susceptible populations, and plate cycling exercise also induced similar changes, which indicated that individual pulmonary artery contractility was the major factor leading to the occurrence of HAPE [42, 43]. This type of patient with hypoxia or high-altitude intolerance can be identified early by exercise load ultrasound. The primary cause of HAPE is hypoxia, which can result in left ventricular diastolic or systolic functional disorder. Left heart functional changes can also trigger pressure-related pulmonary water increase, although studies have demonstrated that no correlation exists between the increased blood flow of the tricuspid valve related to hypoxia or exercise and the changes in E/A, and there was no obvious change in E/E′ under hypoxia or exercise. However, using heart ultrasound, studies have also shown that blood flow velocity across the tricuspid valve increases with the increase in altitude. The ratio of early blood flow velocity to late blood flow velocity (E/A) was significantly lower. The ratio of early and late mitral annulus velocity (Em/Am) was also significantly reduced under tissue Doppler. The increase in trans-tricuspid blood velocity negatively correlated with the decrease in E/A and Em/Am [44]. The left heart's diastolic function was changed, and its degree was closely related to the degree of pulmonary hypertension. With the increase of pulmonary arterial pressure, the pressure of the right heart and interventricular septum has an impact on the diastole of the left heart. Patients with HAPE with different involvement degrees manifest different diastolic function states of the left heart, depending on the degree of right heart involvement caused by pulmonary vasoconstriction.

Pulmonary resection is another common cause of increased pulmonary circulation resistance. The associated PE is termed postpneumonectomy PE (PPE), which was first proposed by Gibbon in 1942. Because of its rapid progression, it often requires mechanical ventilation treatment, and it is difficult to distinguish from ALI or ARDS in clinical practice. The overall incidence of PPE is approximately 7%, and the mortality rate is approximately 12%. One-third of patients can have clinical symptoms within 24 h after surgery, and most patients have dyspnea within 3 days after surgery [45]. The incidence of PPE in patients with overall pneumonectomy is significantly higher than that in patients with partial pneumonectomy. The reduction of the total volume of pulmonary capillaries, pulmonary perfusion, and the increase in pulmonary capillary filtration pressure after pneumonectomy are the key factors leading to its occurrence. Ischemia or reperfusion injury, inflammatory response, endothelial injury, lung overexpansion, and impaired lymphatic drainage are also involved in the pathophysiological process [46, 47]. Intraoperative volume overload, preoperative radiation therapy, infusion of fresh frozen plasma, and intraoperative high-pressure mechanical ventilation are the independent risk factors for PPE [48]. For patients after pneumonectomy, any factor that causes an increase in intrathoracic negative pressure can promote the occurrence of PPE. Deslauriers found that 85% of patients with PPE did not undergo postoperative thoracic closed drainage with water-sealed bottles, and patients who received drainage with a three-chamber balanced drainage system did not experience PP. Alvarez also found similar phenomena [45]. Animal studies have confirmed that intrathoracic pressure suction after pneumonectomy can significantly increase the incidence of PPE, and the occurrence of such PE can be reduced by balanced drainage [49]. These phenomena indicate that in the case of pulmonary overperfusion after pneumonectomy, excessive negative pressure in the chest can increase the trans vascular flow, aggravating the leakage of water across capillaries and causing PE. This necessitates attention to not only the relatively reasonable drainage in the chest but also the factors related to the increase of negative pressure in the chest.

#### 2.2.3. Pleural Cavity Decompression or Negative Pressure

Due to factors such as fluid, gas, and mediastinal or subdiaphragmatic abscess, the pleural cavity can be compressed or incompletely inflated in varying degrees. When these factors are removed, the negative pressure in the pleural cavity restores the lung recruitment and expansion state. There may be PE characterized by hypoxia and dyspnea, which is termedre expansion PE (REPE). The description of REPE appeared more than 150 years earlier. It occurs during drainage of the pleural effusion or pneumothorax or within 24 h. It also occurs in the postresection of thoracic and abdominal cavity lesions and in lung re-expansion during chest surgery, which often occurs on the decompression side. It mostly occurs in the decompression side and rarely occurs in the contralateral or bilateral lung. The overall morbidity and mortality are quite different. The general incidence rate is within 1%, and the mortality rate is 0.1%–20% [50]. The exact pathophysiological mechanism under lying REPE has not been completely elucidated, and it is generally believed to be associated with an excessively rapid decrease of intrapleural pressure, reduction of surface-active substances, release of inflammatory mediators, and generation of oxygen free radicals. Although several studies have suggested that the occurrence of REPE is related to hypoxia and inflammation-related media, an analysis of alveolar fluid components shows that this type of PE is not associated with the increase of inflammation permeability because of the protein component in comparison with plasma [51]. Furthermore, studies show that its occurrence is closely related to hemodynamic changes. First, the characteristics of blood flow in REPE are not changed. In the process of re-expansion, the compressed collapsed lung tissue presents different hypoxia states and vasomotor states; hence, they present low perfusion area and high perfusion area, which has become one of the primary reasons for the increase of pressure pulmonary water [52]. Another cause of the generation of REPE is the rapid change of intrapleural pressure. The rapid decrease of pleural pressure during drainage often indicates that there may be poor lung compliance, visceral pleural compression, and other factors, due to which the lungs cannot undergo full expansion. Excessive transpulmonary pressure and trans vascular pressure, especially for lung tissues with poor compliance, lead to an increase in lung water associated with hydrostatic pressure. When the intrapleural pressure decreases rapidly over −20 cm H_2_O, REPE is easily triggered [53]. The British Thoracic Society recommends that the intrapleural pressure for chest drainage should not exceed −20 cm H_2_O. For patients with REPE, intrapleural fluid or gas is timely administered to reopen the pleural cavity, improving the intrapleural pressure. Partial recovery of atelectasis can rapidly relieve the symptoms of such patients. It further indicates the change of pressure factor plays a role in the occurrence of REPE [51]. Moreover, the increased pleural pressure caused by pleural cavity occupancy may affect the diastolic and systolic function of the left and right ventricles. When the intrapleural pressure is lowered, the diastolic limitation of the heart is relieved and both the blood flow to the heart and the cardiac output are increased [54]. When the diastolic and systolic function of the left heart has obvious obstacles and the left heart cannot withstand the increase of blood flow to the heart, it will aggravate the occurrence of PE [55]. Furthermore, intrathoracic pressure and lung volume have a significant impact on venous return and systolic function. The increase of intrapleural pressure reduces left ventricular transmural pressure, thereby reducing the left ventricular ejection pressure and its upstream pressure. With the decrease of pleural pressure, there is an increase of left ventricular transmural pressure and blood pressure after thoracic drainage. In particular, left ventricular afterload is significantly increased in the case of significantly increased intrathoracic negative pressure, resulting in decreased left ventricular function and PE, especially in patients with left ventricular lesions [56]. This suggests the need to perform echocardiography to identify left cardiac function during pleural decompression in high-risk patients to determine the potential risk for REPE.

Another type of hemodynamically altered PE, which is closely related to changes in intrathoracic negative pressure, is negative pressure PE (NPPE) which occurs in various causes of excessive intrathoracic negative pressure. This PE is common in obstruction of the airway which a variety of causes result in, also known as post obstructive PE, such as spasms after extubating, the conjugate neck, epiglottis, airway inhalation of foreign bodies, secretion, serious hiccup, laryngitis, upper airway, and mediastinal tumor, Ludwig angina, obstructive sleep apnea, severe asthma, tracheal intubation or laryngeal mask bite, and so on. In 1977, Oswalt first described NPPE as a serious complication of airway obstruction [57], which can lead to pulmonary capillary rupture and pulmonary hemorrhage in more severe cases [58]. Forced inhalation to overcome airway resistance can produce a negative intrathoracic pressure of up to −140 cm H_2_O, causing a significant increase in blood flow from the venous return to the right heart, whereas the backload of the left heart is significantly increased due to increased cross-wall pressure. The reduction of cardiac output and the increase of pulmonary venous pressure lead to a significant increase in the hydrostatic pressure of pulmonary circulation. Moreover, the negative pressure in the chest can be transmitted to the lung tissue, causing an increase in the gradient of trans vascular hydrostatic pressure, which causes the water inside the blood vessels to enter into the alveolar cavity. In addition, hypoxia induces sympathetic reflex and causes peripheral vascular contraction, and the blood flow from the systemic circulation to the pulmonary circulation is redistributed. Hypoxia also leads to heterogeneous contraction of pulmonary vessels, which further causes overperfusion of increased blood flow, resulting in NPPE occurrence. The occurrence of NPPE is closely related to the degree of intrathoracic negative pressure and the body's reactivity and sympathetic activation, which explains why NPPE is more likely to occur in healthy men [59].

## 3. Treatment of Pulmonary Oedema

### 3.1. Clinical Treatment

The most common symptom of pulmonary edema is dyspnoea, and patients with cardiogenic pulmonary edema present irritability, choking, and cyanosis, and in severe cases, coma, along with the corresponding clinical manifestations of the primary disease [60]. Dyspnoea, seated breathing, irritability, and asphyxia are the typical symptoms of pulmonary edema and may be accompanied by other symptoms, such as coughing in the early stages of cardiogenic pulmonary edema, coughing up pink frothy sputum in severe cases and increased or normal blood pressure in the early stages, which may cause cardiogenic shock [61]. The principles of treatment for pulmonary edema are correction of the primary cause of pulmonary edema, and respiratory support to improve patient oxygenation [62]. Non-invasive positive pressure ventilation is the first line of treatment to improve cardiogenic pulmonary edema and correct hypoxemia; in patients, who are already mechanically ventilated, a lung-protective ventilation strategy needs to be implemented to avoid further damage to alveolar epithelial cells and vascular endothelial cells from mechanical ventilation [63]. Due to the drastic individual differences, there is no unifying medication. Apart from the commonly used over-the-counter drugs, the most appropriate medication should be selected under the guidance of a doctor with full consideration of individual conditions. Diuretics and vasodilators should be applied to reduce the anterior-posterior cardiac load and pulmonary capillary pressure, thereby reducing the patient's pulmonary edema; doctors should apply appropriate cardiac strengthening drugs to enhance the patient's myocardial contractility; antibiotic therapy should be reasonably applied to control infection, and glucocorticoids to inhibit the inflammatory response and promote the reduction of edema [64–66].

### 3.2. The Use of Chinese Medicine in the Treatment of Pulmonary Oedema

The treatment of pulmonary edema is fast with Western medicine and has a high success rate of resuscitation, but timely treatment with traditional Chinese medicine (TCM) can significantly shorten the course of the disease [67]. According to anatomy, the etiology of pulmonary edema can be divided into two categories: cardiac and noncardiac, and therefore the TCM treatment of pulmonary edema is carried out from these two aspects [68]. As far as cardiogenic acute pulmonary edema is concerned, its onset is rapid, and the TCM syndrome differentiation is that qi is deprived of yang, and phlegm is forced into the lung [69]. According to reports, the combination of ginseng and aconite can promote blood circulation, improve microcirculation disorders, expand and strengthen the heart, and improve symptoms of heart failure; cinnamon contains cinnamon oil, which has central and terminal vasodilator effects and can enhance blood circulation [70]; Helizao Xiefei Decoction has the functions of purging the lung and relieving asthma, eliminating phlegm, strengthening the heart, reducing the blood return to the heart and improving the pulmonary ventilation function [71]. Traditional Chinese medicines such as astragalus, poria, atractylodes, psyllium, coix seed, gourd, and atractylodes can play a certain role in relieving acute symptoms of pulmonary edema (such as chest tightness, cough, and asthma) [72, 73]. Modern pharmacological experimental studies have found that these diuretics can reduce the resistance of the arteries and veins, allowing a venous return to flow smoothly and reducing pulmonary hypertension, so that the patient's edema, coughing, chest tightness, and a series of other clinical symptoms can be relieved [74]. During acute attacks, the effect is more rapid if Chinese medicine for the spleen is used together with diuretic western medicine [75]. However, strengthening the spleen tends to damage the kidneys, i.e., too many diuretic Chinese and Western medicines can easily lead to damage to the patient's positive energy, fatigue, and depression. Therefore, while strengthening the spleen and diuresis, TCM practitioners should also tonify the patient's kidney essence [76]. For those, who favor kidney yin deficiency, use Liou Wei Di Huang Wan and Er Zhi Wan to tonify kidney yin; for those, who favor yang deficiency, use Gui Bai Di Huang Wan or Jin Kui Kidney Qi Wan to warm up kidney yang [77–79].

## 4. Conclusions

PE is a serious stage of acute and chronic heart failure, and it is generally described as the inevitable result of increased left ventricular filling pressure. When the cardiac afterload increases or the left ventricular function is impaired, the left ventricular discharge decreases, and the left ventricular end-diastolic pressure increases. The left atrial pressure then increases, which elevates the pulmonary capillary hydrostatic pressure. Hence, it is basically stated that PE is caused by the mismatch of the stroke volume of the left and right ventricles. According to the Frank–Starling law, one of the important factors in the development of PE is that the capillary hydrostatic pressure of the pulmonary circulation is significantly increased. The capillary hydrostatic pressure is primarily maintained by the pressure generated by the right heart, so the right heart plays a vital role in the development of PE. Normal pulmonary circulation is a system of high flow, low resistance, and low pressure under normal conditions. Any factor that causes abnormal pulmonary circulation will cause a mismatch between the right heart and pulmonary circulation flow, resulting in PE. Therefore, the right heart plays an important role in the development of PE.

## Figures and Tables

**Table 1:** Key points of the category of right heart-associated PE.

*Increased right heart flow*	
Extravascular compression	Peripheral venous contraction is caused by various reasons.
Intravascular compression	The relative or absolute overload of blood vessel volume.
Cardiac pressurization	The left heart function is weakened or the enhancement of right cardiac systolic activity.
Cardiac decompression	The decompression of the pericardium or pleural cavity.

*Abnormal pulmonary circulation*	
Obstructive factors	Pulmonary embolism
Resistance factors	Pulmonary arterial hypertension
Pleural cavity decompression or negative pressure	The negative pressure in the pleural cavity restores the lung recruitment and expansional state.

## Data Availability

The datasets used and analyzed during the current study are available from the corresponding author on reasonable request.
